The article "The effect of lower limb rehabilitation gymnastics on postoperative rehabilitation in elderly patients with femoral shaft fracture: A retrospective case-control study" was published in 2016. Journal: Medicine (Baltimore).

# The effect of lower limb rehabilitation gymnastics on postoperative rehabilitation in elderly patients with femoral shaft fracture: A retrospective case-control study

**DOI:** 10.1097/MD.0000000000004548

**Published:** 2016-08-19

**Authors:** Si-Dong Yang, Sheng-Hua Ning, Li-Hong Zhang, Ying-Ze Zhang, Wen-Yuan Ding, Da-Long Yang

**Affiliations:** a Department of Spinal Surgery, The Third Hospital of Hebei Medical University, Ziqiang Road, Shijiazhuang; b Department of Orthopaedic Surgery, Longyao County Hospital, Longyao; c Hebei Provincial Key Laboratory of Orthopaedic Biomechanics, Shijiazhuang, Hebei Province, China.

**Keywords:** elderly femoral shaft fracture, lower limb rehabilitation gymnastics, orthopedic nursing, postoperative rehabilitation, prognosis

## Abstract

The purpose of this study was to explore the effect of lower limb rehabilitation gymnastics on postoperative rehabilitation in elderly patients with femoral shaft fracture after undergoing intramedullary nail fixation surgery.

We collected medical records of elderly patients aged ≥ 60 years with femoral shaft fracture between 03/2010 and 03/2015 in Longyao County Hospital. Totally, 160 patients were identified and divided into the intervention group (n = 80) and the control group (n = 80). During the postoperative period, the intervention group received lower limb rehabilitation gymnastics treatment for 3 months, but the control group did not. All patients were routinely asked to return hospital for a check in the 1st postoperative week, as well as the 2nd week, the 1st month, and the 3rd month, after surgery. The clinical rehabilitation effect was evaluated by checking lower limb action ability, detecting the lower limb deep venous thrombosis (DVT), scoring muscle strength of quadriceps and visual analog scale (VAS) score, and performing satisfaction survey.

At the 1st week and 2nd week after surgery, the clinical rehabilitation effect in the intervention group was better regarding lower limb action ability, lower limb DVT, muscle strength of quadriceps, VAS score, and patient satisfaction, as compared with the control group. However, there was no significant difference at the 1st month and the 3rd month after surgery when comparing the intervention group to the control group.

In the early postoperative stage, lower limb rehabilitation gymnastics can effectively improve the recovery of lower limb function, beneficial to reducing postoperative complications such as lower limb DVT and muscle atrophy, and increasing patient satisfaction rate.

## 1 Introduction

Worldwide, road injuries cause >1.3 million deaths and many more disabilities annually, disproportionately affecting the young and the poor.^[1]^ Approximately 1 in 10 road injuries involves a femoral shaft fracture that is most effectively treated with surgery.^[1]^ To our knowledge, intramedullary nail fixation is the most popular surgical method to perform an operation for the patients with femoral shaft fracture. As the population ages, the incidence of femoral shaft fractures in elder patients seems to increase.^[2]^ Thus, knowledge of the results of treatment in this age group is important to the orthopedic surgeon.

The article "The effect of lower limb rehabilitation gymnastics on postoperative rehabilitation in elderly patients with femoral shaft fracture: A retrospective case-control study" was published in 2016. Journal: Medicine (Baltimore).

It has been reported that intramedullary nailing of femoral shaft fractures in patients over the age of 60 years is an effective method of treatment.^[2]^ However, elder patients suffering from femoral shaft fractures are very different from those younger patients with the same disease. Elder patients may experience longer on-bed time in a hospital after being performed an operation of intramedullary nailing fixation of femoral shaft fractures, as compared to younger patients. In addition, it is another long term for the elderly patients to recover from an operation trauma, due to the aged body and weak physical function. Therefore, during that period, postoperative complications, such as deep venous thrombosis (DVT) and lower limb muscle atrophy, are more likely to occur and increase. However, few studies have reported on this problem existing in the process of recovery from femoral shaft fracture after surgery.

Clinically, we have often asked the elderly patients with femoral shaft fracture to perform lower limb rehabilitation gymnastics as a prophylaxis of postoperative complications. Thus, the aim of this study is to explore whether this method (lower limb rehabilitation gymnastics) is effective on postoperative rehabilitation in elderly patients with femoral shaft fractures.

## 2 Patients and methods

### 2.1 Ethics statement

Regarding the present study, there is no need to obtain informed consent from patients as this is a retrospective case-control study and all the data were collected and analyzed anonymously without any potential harm to patients.

### 2.2 Patients and inclusion criteria

We collected medical records of elderly patients aged > / = 60 years with femoral shaft fracture between 03/2010 and 03/2015 in Longyao County Hospital. As Fig. 1 showed, there were totally 242 cases, but 160 patients were identified and admitted to this study, among which 96 were males and 64 were females. The average age was 67 ± 6 years old. Among them, no cases in the intervention group or in the control group were nonunions. Also, no patients were infected after surgery. Inclusion criteria of the present study were as follows: (1) no history of other fractures were on the same limb; (2) no history of other operations were on the same limb; (3) no neuromuscular disease were on the same limb; (4) no pathologic fracture existed; (5) all patients have undergone intramedullary nail fixation surgery for femoral shaft fracture; (6) all the patients have been excluded from DVT by preoperative ultrasonography. Patients who did not have regular follow-up visits or had systemic disorders were excluded.

The article "The effect of lower limb rehabilitation gymnastics on postoperative rehabilitation in elderly patients with femoral shaft fracture: A retrospective case-control study" was published in 2016. Journal: Medicine (Baltimore).

**Figure 1:** Flow diagram used for patient selection.

### 2.3 Intervention methods

The patients according to the treatment during that period were divided into the intervention group or the control group, 80 cases in each group. In the intervention group, there were 45 males and 35 females. In the control group, there were 51 males and 29 females. During the perioperative period, both the intervention group and the control group received the same routine nursing care and drug treatment including low-molecular-weight heparin (LMWH) after surgery. During the postoperative period, the intervention group received lower limb rehabilitation gymnastics treatment for 3 months, but the control group did not. The lower limb rehabilitation gymnastics was performed as follows. In the first section, let the patients lie flat with relaxation. In the second section, let them centripetally massage double lower limbs for 5 minutes. In the third section, ankle pump movement, let double foot try to flex or extend for 5 seconds, repeating 50 times per section, 3 sections each day. In the fourth section, knee-pressing motion, keeping legs straight, try to press knees down for 10 seconds, repeating 20 times per section, 3 sections each day. In the fifth section, let quadriceps stay static contraction and double lower limbs unbend; then try to let foot stand and lower limbs press down on bed, maintaining for 10 seconds, repeating the movement 20 times per section, 3 sections each day. In the last section, bend your knees and hip, and make the double knee joints flex for 30 degrees, keeping relaxed, repeating 20 times per section, 3 sections each day.

### 2.4 Evaluation of rehabilitation effect

All patients were routinely asked to return hospital for a check in the 1st postoperative week, as well as the 2nd week, the 1st month, and the 3rd month, after surgery. The clinical rehabilitation effect was evaluated by checking lower limb action ability, detecting the lower limb DVT, scoring muscle strength of quadriceps and visual analog scale (VAS) score, and performing satisfaction survey. Regarding checking lower extremities action ability, patients were asked to complete some regular movements. It was regarded as excellent when >90% movements were completed, good for 70% to 90%, poor for <70%. As for evaluating muscle strength of quadriceps, the Lovett muscle strength classification standard was applied. In addition, the satisfaction survey was classified into 3 grades, very satisfied, satisfied, and dissatisfied.

The article "The effect of lower limb rehabilitation gymnastics on postoperative rehabilitation in elderly patients with femoral shaft fracture: A retrospective case-control study" was published in 2016. Journal: Medicine (Baltimore).

### 2.5 Statistical analyses

Statistical analyses were performed using SPSS for Windows, version 18.0 (SPSS Inc.). All measurement data are presented as the mean ± SD (standard deviation) when data satisfied criteria for normality with *P* > 0.10. Otherwise, it should be presented as median (interquartile range, IQR). When data satisfied criteria for normality and homogeneity of variance, statistical analysis between groups was performed using Student's *t* test. Otherwise, statistical analysis was performed using the Mann–Whitney *U* test. For count data, the chi-square test was used for data analysis. Values for *P* < 0.05 were regarded as significant with 2-tailed tests.

## 3 Results

### 3.1 Lower limb action ability

As shown in Table 1, during the first 2 weeks after surgery, lower limb action ability in the intervention group was better than that in the control group (χ^2^ = 4.98, *P* = 0.026;χ^2^ = 10.88, *P* = 0.001, respectively). However, there was no significant difference on the time points of the 1st month and the 3rd month after surgery when comparing the intervention group with the control group regarding lower limb action ability (χ^2^ = 0.23, *P* = 0.633).

**Table 1:** Comparison of intervention group with control group regarding lower limb action ability.

### 3.2 Lower limb DVT

As shown in Table 2, during the first 2 weeks after surgery, lower limb DVT in the intervention group was less than that in the control group (χ^2^ = 4.44, *P* = 0.035;χ^2^ = 5.74, *P* = 0.017, respectively). As well, lower limb DVT in the intervention group was less than that in the control group on the time point of the 1st month after surgery (χ^2^ = 5.33, *P* = 0.021). However, there was no significant difference on the time point of the 3rd month after surgery when comparing the intervention group with the control group regarding lower limb DVT (Fisher Exact Test, *P* = 0.443).

**Table 2:** Comparison of intervention group with control group regarding lower limb deep venous thrombosis (DVT).

### 3.3 Muscle strength of quadriceps

As shown in Table 3, during the first 2 weeks after surgery, the patients with grade IV and grade V of muscle strength in the intervention group were more than those in the control group (χ^2^ = 10.00, *P* = 0.002;χ^2^ = 5.96, *P* = 0.015, respectively). However, there was no significant difference on the time points of the 1st month and the 3rd month after surgery when comparing the intervention group with the control group.

The article "The effect of lower limb rehabilitation gymnastics on postoperative rehabilitation in elderly patients with femoral shaft fracture: A retrospective case-control study" was published in 2016. Journal: Medicine (Baltimore).

**Table 3:** Comparison of intervention group with control group regarding muscle strength of quadriceps (Lovett muscle strength classification standard).

### 3.4 VAS score

As shown in Table 4, during the first 2 weeks after surgery, the VAS score in the intervention group was less than that in the control group (*t* = 6.99, *P* < 0.001; *t* = 3.00, *P* = 0.003, respectively). However, there was no significant difference on the time points of the 1st month and the 3rd month after surgery when comparing the intervention group with the control group regarding the VAS score (*t* = 1.40, *P* = 0.163; *t* = 0.82, *P* = 0.420, respectively).

**Table 4:** Comparison of intervention group with control group regarding the VAS score.

### 3.5 Satisfaction survey

As shown in Table 5, during the first 2 weeks after surgery, the satisfaction rate in the intervention group was higher than that in the control group (χ^2^ = 10.00, *P* = 0.002;χ^2^ = 6.94, *P* = 0.008, respectively). However, there was no significant difference on the time points of the 1st month and the 3rd month after surgery when comparing the intervention group with the control group regarding the satisfaction rate (Fisher Exact Test, *P* = 0.443, *P* > 0.99, respectively).

**Table 5:** Comparison of intervention group with control group regarding satisfaction survey.

## 4 Discussion

It is well known that femoral shaft fracture in the elderly is often caused by falling down, an accident, violence, and torsion. And it usually results in some clinical symptoms including limitation of motion and hip pain. Additionally, it has been reported that osteoporosis is a risk factor associated with femoral shaft fracture,^[3]^ which may result from the reduction of bone cells, change of bone microstructure, the decrease of both bone strength, and bone mineral density. Currently, most studies on intramedullary nailing fixation for femoral shaft fracture are about patients >60 years old, which have well demonstrated that intramedullary nailing fixation is an established and accepted surgical procedure, but data on the results of this treatment on the patients >60 years old are not many.^[2,4]^ It has been determined that the outcome of intramedullary nailing fixation for femoral shaft fracture in elderly patients is also acceptable.^[4]^ It is of no significant difference regarding the clinical outcomes of intramedullary nailing fixation treatment between the elderly patients and younger patients, except more symptoms found in the elderly.^[4]^

It is true that elder patients suffering from femoral shaft fractures are very different from those younger patients with the same disease. Elder patients are believed to experience longer hospital time after undergoing an operation of intramedullary nailing fixation of femoral shaft fractures compared to younger patients. In addition, it is another long term for the elderly patients to recover from an operation trauma, due to the aged body and their own weak physical function. Therefore, during that period, postoperative complications, such as DVT and lower limb muscle atrophy, are more likely to occur and increase. However, few studies have discussed on this existing topic regarding the prophylaxis of postoperative complications, especially in the process of recovery from femoral shaft fracture after surgery.

The article "The effect of lower limb rehabilitation gymnastics on postoperative rehabilitation in elderly patients with femoral shaft fracture: A retrospective case-control study" was published in 2016. Journal: Medicine (Baltimore).

In clinical situations, we often asked and guided the patients to do exercise after an operation according to the procedures of lower limb rehabilitation gymnastics. But we did not assess the effect then. Herein, this study has been designed and performed to evaluate the effect of lower limb rehabilitation gymnastics on the functional recovery and complications developed during the process of functional recovery. As a consequence, in the early stage after surgery (during the first 2 weeks), lower limb action ability, muscle strength of quadriceps, and patient satisfaction rate are better in the intervention group when compared to the control group. Besides, lower limb DVT and VAS score are less in the intervention group as compared to the control group. However, there is no significant difference between the 2 groups regarding the above items evaluated in the later stage (on the timepoint of the 1st and the 3rd month).

A variety of factors such as age, prefracture function and health status, fracture type, pain, anemia, muscle strength, and the early mobility level have been shown to influence patient outcome.^[5]^ Thus, the outcome of patients with hip fracture is considered multifactorial^[5]^ and can therefore not be related to just 1 or 2 single factors. Additionally, patients are at risk of decreased physical function,^[6–8]^ new injurious falls and fractures,^[9,10]^ and increased need of supportive care.^[11]^

With respect to recovery after a hip fracture, early mobilization ^[12–14]^ and extended physical therapy including strength training implemented 6 weeks after fracture seem to promote recovery of physical function.^[15]^ It is also found that after a hip fracture, most recovery of the function happens within the first 3 months, although some functional activities continue recovering over the first year.^[8]^ Hence, that is why the endpoint of the present study is limited to the 3rd month after surgery. In reality, some studies^[16–18]^ previously reported have supported the point of view that early exercise or mobilization can reduce the risk of developing lower limb DVT after an operation. And early mobilization in patients with acute deep vein thrombosis does not increase the risk of a symptomatic pulmonary embolism.^[16]^ The incidence of early postoperative DVT in legs was reduced by 77% after prevention by passive exercise of leg during surgery.^[17]^ There is a reduction in risk of postoperative thromboembolism with early ankle movement.^[18]^

Regarding the VAS score reported in the current study, it has been found that lower limb rehabilitation gymnastics does not increase hip pain, but relieves postoperative pain to a certain degree. Previously, Kronborg et al^[19]^ has ever reported that progressive knee-extension strength training of the fractured limb commenced in the acute ward seems feasible, and may reduce strength asymmetry between limbs without hip pain interfering. Both of the 2 studies reported here believe that early intervention postoperatively do not increase any pain to the elderly patients. Of note, most of previous studies and ours have been designed that rehabilitation programs are based only on mobility activities in the early postoperative stage. However, Ariza-Vega et al has claimed that rehabilitation programs cannot be based only on mobility activities, the recovery of other daily living activities should also be included.^[8]^ It seems more reasonable when we consider intervening in the postoperative recovery of the elderly patients from femoral shaft fractures.

The article "The effect of lower limb rehabilitation gymnastics on postoperative rehabilitation in elderly patients with femoral shaft fracture: A retrospective case-control study" was published in 2016. Journal: Medicine (Baltimore).

Compared to younger patients, elderly patients are poorer in terms of physical condition and postoperative recovery ability. Thus, it is of special significance to concentrate on the present topic related to femoral shaft fracture in the elderly patients. Surely, this study has indicated very important clinical significance. However, this work also has some limitations. First, as a retrospective single-center case-control study, it lacks extensive representativeness. Second, we have not applied blind methods throughout the study. Third, the sample size of patients included in the study is not large enough. So future research should strive to overcome these shortcomings, provide more reliable clinical research data. It is best to be a large sample, prospective, multicenter, randomized, controlled study, with blind methods applied.

In conclusion, in early postoperative stage, lower limb rehabilitation gymnastics can effectively improve the recovery of lower limb function, beneficial to reducing postoperative complications such as lower limb DVT and muscle atrophy, and increasing patient satisfaction rate, as for the elderly patients suffering from femoral shaft fractures with intramedullary nailing fixation.
